# Restoration of Mal overcomes the defects of apoptosis in lung cancer cells

**DOI:** 10.1371/journal.pone.0227634

**Published:** 2020-01-24

**Authors:** Li-Tao Yang, Fei Ma, Hao-Tao Zeng, Miao Zhao, Xian-Hai Zeng, Zhi-Qiang Liu, Ping-Chang Yang

**Affiliations:** 1 ENT Institute, Research Center of Allergy & Immunology, Shenzhen University School of Medicine, Shenzhen, China; 2 Guangdong Provincial Key Laboratory of Regional Immunity and Diseases, Shenzhen, China; Chung Shan Medical University, TAIWAN

## Abstract

**Background and aims:**

Cancer is one of the life-threatening diseases of human beings; the pathogenesis of cancer remains to be further investigated. Toll like receptor (TLR) activities are involved in the apoptosis regulation. This study aims to elucidate the role of Mal (MyD88-adapter-like) molecule in the apoptosis regulation of lung cancer (LC) cells.

**Methods:**

The LC tissues were collected from LC patients. LC cells and normal control (NC) cells were isolated from the tissues and analyzed by pertinent biochemical and immunological approaches.

**Results:**

We found that fewer apoptotic LC cells were induced by cisplatin in the culture as compared to NC cells. The expression of Fas ligand (FasL) was lower in LC cells than that in NC cells. FasL mRNA levels declined spontaneously in LC cells. A complex of FasL/TDP-43 was detected in LC cells. LC cells expressed less Mal than NC cells. Activation of Mal by lipopolysaccharide (LPS) increased TDP-43 expression in LC cells. TDP-43 formed a complex with FasL mRNA to prevent FasL mRNA from decay. Reconstitution of Mal or TDP-43 restored the sensitiveness of LC cells to apoptotic inducers.

**Conclusions:**

LC cells express low Mal levels that contributes to FasL mRNA decay through impairing TDP-43 expression. Reconstitution of Mal restores sensitiveness of LC cells to apoptosis inducers that may be a novel therapeutic approach for LC treatment.

## Introduction

Lung cancer (LC) is one of the leading causes of human death in the world [1]. The symptoms of LC are not specific, and may include weight loss, cough, bloody sputum, and feeling tired all the time. The pathogenesis of LC is unclear; the oncogene activation, inactivation of tumor suppressor genes, and gene mutations may contribute to the development of LC [2]. The LC therapeutic efficacy is currently unsatisfactory [3]. Therefore, it is necessary to further investigate the pathogenesis of LC and invent novel and effective remedies for LC treatment.

Therapeutic approaches for LC mainly include surgery, chemotherapy, radiotherapy and biotherapy. Besides surgery, one of the mechanisms of these therapies is to induce cancer cell apoptosis [4]. Therefore, the dysregulation of apoptosis in cancer cells is a large obstacle in LC treatment [5]. Apoptosis is a physiological process by which the senescent and unwanted cells are eliminated; it is also called programmed cell death [6]. Apoptosis is initiated by intrinsic events or/and extrinsic events. Some regulatory factors for apoptosis have been recognized; e.g., Fas/Fas ligand and caspases involve initiating apoptosis, while some others, e.g., Bcl-2 family, inhibit apoptosis [7]. Over-inhibition of apoptosis may result in the defects of apoptosis in the cell [7]. Although research of apoptosis advanced rapidly in the recent years, yet, factors of inducing the defects of apoptosis in cancer cells remain to be further elucidated.

Microbial factors, such as lipopolysaccharide (LPS), can regulate the process of apoptosis [8]. The Toll like receptors (TLR) mediate microbial stimuli to induce a series of bioactivities in the body [9]. Myeloid differentiation factor 88 (MyD88) and Mal (MyD88-adapter-like) are the critical components in the TLR signal transduction pathway of all TLRs (except TLR3). Published data indicate that Mal is involved in the process of apoptosis [10]; while whether Mal is associated with the pathogenesis of the defects of apoptosis in cancer is unclear.

The RNA decay is associated with the pathogenesis of cancer [11]; it is a physiological phenomenon that eliminates those RNAs not properly processed [12]. Prior to translation, RNA-binding proteins bind to the poly (A) nucleotide tail of RNA to prevent RNA from degradation to regulate RNA production. If the poly (A) tail does not add properly, the RNA may be degraded quickly, result in RNA decay [13]. TAR DNA-binding protein (TDP-43) is an essential DNA- and RNA-binding protein [14]. TDP-43 controls gene expression through RNA processing, such as regulation of splicing. TDP-43 is localized in the cytoplasmic stress granules, which may relate to pathological activities [15]. It is recognized that TDP-43 associates with the pathogenesis of cancer [16]. Yet, whether TDP-43 is involved in the development of the defects of apoptosis in LC is unclear.

Therefore, in this study, we collected LC samples from surgically removed LC tissues. The defects of apoptosis in LC cells were recognized, which was associated with the deficiency of TDP-43 in LC cells.

## Materials and methods

The experimental procedures were approved by the Human Ethic Committee at Shenzhen University (180003).

### Reagents

Antibodies of Fas (sc-8009), Fas ligand (sc-71096), Toll-like receptor-4 (sc-293072), MyD88 (sc-136970), Mal (sc-390687), TDP-43 (sc-100871) and shRNA kit of Mal, TLR4 (sc-40260) and TDP-43 (sc-154072) were purchased from Santa Cruz Biotech (Santa Cruz, CA). Anti-KRT8 antibody (ab191208) was purchased from abcam (Cambridge, MA). Lipopolysaccharides, fluorometric assay kits for caspase 8 and caspase 3, cisplatin, annexin v kit (APOAF-20TST) and RNA-immunoprecipitation reagents/materials were purchased from Sigma Aldrich (St. Louis., MO). Reagents and materials for RT-qPCR and Western blotting were purchased from Invitrogen (Carlsbad, CA).

### Human subjects

This study was carried out in the Research Center of Allergy & Immunology at Shenzhen University. Patients with LC were recruited into this study at the affiliated hospitals of Shenzhen University (Shenzhen, China) from January 2018 to April 2019. The diagnosis and management of LC were carried out by our surgeons and pathologists following our routine procedures. The criteria of recruiting LC patients include: (1) LC; (2) not under specific LC therapies yet; (3) the LC was to be treated by surgery. The demographic data of patients are presented in Table 1. Patients with any of the following conditions were excluded from this study, including under treatment with immune suppressors, allergic diseases, autoimmune diseases and severe organ diseases. A written informed consent was obtained from each human subject.

**Table 1:** Demographic data of patients with lung cancer.

Items	
Male	10 (55.6%)
Female	8 (44.4%)
Age	56.5 ± 8.6 years
Cancer type	NSCLC
Recurrence	0

NSCLC: Non-small cell lung cancer.

### Preparation of LC cells and normal control (NC) cells

Surgically removed LC tissue was collected in the operation facilities of our hospital. LC tissue and marginal normal tissue (proved by pathologists with histology procedures) were cut into small pieces, incubated with collagenase IV (1 mg/ml) at 37°C with mild agitation. Single cells were filtered through a cell strainer (70 μm first, then 40 μm) and collected by centrifugation (1,000 g x 5 min). LC cells were purified from single cells by magnetic cell sorting (MACS), in which the KRT8, an epithelial cytoskeleton gene, was used as the LC marker and NC epithelial cell marker; the cells were isolated by flow cytometry cell sorting. NC cells and LC cells isolated from individual subjects were processed and analyzed separately.

### Cell culture

NC cells and LC cells were cultured in DMEM. The medium was supplemented with antibiotics (streptomycin and penicillin), fetal calf serum and glutamine. The medium was changed daily. Cell viability was greater than 99% as assessed by Trypan blue exclusion assay.

### Induction of apoptosis in NC cells and LC cells

NC cells and LC cells were prepared and cultured in the presence of cisplatin at 10 μM/ml for 48 h. The cells were analyzed by flow cytometry.

### Assessment of apoptotic cells

Cells were stained with propidium iodide (5 μg/ml) and annexin v reagent following the manufacturer's instructions. The cells were analyzed with a flow cytometer (FACSCanto II). Data were analyzed with software package flowjo. Data from none stained cells were used as gating references.

### Real-time quantitative RT-PCR (RT-qPCR)

Cells were collected from relevant experiments. Total RNA was extracted from the cells with TRIzol reagents. The cDNA was synthesized from RNA with a reverse transcription reagent kit following the manufacturer's instructions. The samples were amplified in a qPCR device with the SYBR Green Master Mix in the presence of relevant primers, including TLR4 (gtgcctccatttcagctctg and caaagatacaccagcggctc), FasL (cagcagcccttcaattaccc and gctgtggttccctctcttct), Mal (gtctgcgcggagtctgag and gagccactcacaaactcaaaga) and TDP-43 (gcagatgatcagattgcgca and aacgcaccaaagttcatccc). Data were processed using the 2^-ΔΔCt^ method with pooled RNA of NC sample (not stimulated) as a control. The results are presented as relevant change.

### Protein extraction

Cells were collected from relevant experiments and lysed with a lysis buffer (10 mM HEPES; 1.5 mM MgCl2; 10 mM KCl; 0.5 mM DTT; 1 mM EDTA; 0.05% NP40). The lysates were centrifuged for 10 min at 13,000 g. Supernatant was collected and used as cytosolic protein extracts. The pellets were lysed with a nuclear lysis buffer (5 mM HEPES; 1.5 mM MgCl_2_SO_4_; 4.6 M NaCl; 0.2 mM EDTA; 0.5 mM DTT; 26% glycerol) and centrifuged for 10 min at 13,000 g. Supernatant was collected and used as nuclear protein extracts. The procedures were performed at 4°C.

### Western blotting

Cells were harvested from relevant experiments. Total proteins were extracted from cells with protein extraction buffer (10 mM HEPES; 1.5 mM MgCl2; 10 mM KCl; 0.5 mM DTT; 1 mM EDTA; 0.05% NP40), fractioned by SDS-PAGE, and transferred onto a PVDF membrane. The membrane was blocked with 5% skim milk for 30 min, incubated with the primary antibodies of interest overnight at 4°C, washed with TBST (Tris-buffered saline containing 0.1% Tween 20) 3 times, incubated with the second antibodies (labeled with peroxidase) for 2 h at room temperature and washed 3 times with TBST. Immunoblots on the membrane were developed with enhanced chemiluminescence and photographed with an imaging device.

### RNA immunoprecipitation

Cells were harvested from relevant experiments and radiated with UV for 15 min to cross-link mRNA and protein. The cells were lysed with a lysis buffer (10 mM HEPES; 1.5 mM MgCl2; 10 mM KCl; 0.5 mM DTT; 1 mM EDTA; 0.05% NP40). The lysates were precleared by incubating with protein G agarose beads for 2 h. The beads were removed by centrifugation at 5,000 g for 10 min. The supernatant was collected and incubated with antibodies of interest or isotype IgG overnight. The immunocomplexes in the samples were precipitated by incubating with protein G agarose beads for 2 h. The beads were collected by centrifugation at 5,000 g for 10 min. Complexes of RNA/proteins were eluted from the beads with an eluting buffer. RNA was extracted from the samples with an RNA extracting reagent kit following the manufacturer's instructions. The RNA was analyzed by RT-qPCR and the proteins were analyzed by Western blotting. The procedures were performed at 4°C.

### Assessment of caspase activities

Caspase 8 and caspase 3 activity was measured in NC cells and LC cells (1×10^6^/ml) by monitoring cleavage of the caspase 8- or caspase 3-specific fluorogenic substrate according to the manufacturer’s instructions.

### RNA interference (RNAi)

Mal or TDP-43 expression was knocked down in NC cells or LC cells by RNAi with a Mal RNAi reagent kit or TDP-43 reagent kit following the manufacturer’s instructions. The effect of RNAi was assessed by Western blotting 48 h later.

### Reconstitution of Mal or TDP-43 in LC cells

Mal expression or TDP-43 expression was reconstituted in LC cells by transfecting LC cells with Mal-expressing plasmids (or control plasmids) or TDP-43-expressing plasmids (or control plasmids) (the plasmids were provided by Sangon Biotech (Shanghai, China) following the manufacturer’s instructions. The effects of reconstitution were assessed by Western blotting 48 h after transfection.

### Statistics

The difference between the 2 groups was determined by Student *t* test. ANOVA was employed for multiple comparisons followed by Dunnett’s test or Bonferroni test. Correlation of data between the two groups was determined by Pearson Correlation assay. P<0.05 was considered statistical significance.

## Results

### Apoptotic defects in LC cells are positively correlated with FasL expression

LC cells were isolated from surgically removed LC. Normal control (NC) cells were isolated from the marginal none cancer tissues (proved by a pathologist). The cells were exposed to cisplatin (an apoptosis inducer; saline was used as a control agent) in the culture and analyzed by flow cytometry. We found that only a smaller number of apoptotic cells was induced in LC cells as compared to that in NC cells (Fig 1A and 1B), indicating that LC cells have the defects of apoptosis. Since FasL plays a critical role in the induction of apoptosis [17], the FasL expression in the cells was evaluated. The FasL expression was lower in LC cells than that in NC cells (Fig 1C and 1D). The levels of p53, Bax, Fas, caspase 3 and caspase 8 were not significantly different between LC samples and NC samples (S1 Fig). A positive correlation was identified between the FasL expression and the apoptotic cell number (Fig 1E and 1F). The results indicate that LC cells express less FasL that may contribute to the defects of apoptosis in LC cells.

**Fig 1:** Apoptotic defects in LC cells. The lung cancer (LC) tissues were collected from LC patients (n = 18). LC cells and NC cells (marginal normal tissues; proved by a pathologist) were isolated from the tissues and exposed to cisplatin or saline (vehicle, used as a control) in the culture for 48 h to induce apoptosis. The cells were analyzed by flow cytometry, RT-qPCR and Western blotting. A, gated cells are apoptotic cells. B, summarized data of apoptotic cells in panel A. C, FasL mRNA levels. D, FasL protein levels. E-F, positive correlation between FasL mRNA and apoptotic cells after exposing to cisplatin. Data of bars are presented as mean ± SEM. Each dot in bars presents data obtained from one sample. Statistics: *t* test.

### FasL mRNA spontaneously decay in LC cells

Since RNA decay is a physiological phenomenon in the cell [12], data of Fig 1 imply FasL mRNA may decay spontaneously in LC cells. To test the inference, NC cells and LC cells were cultured in complete DMEM. The cells were stimulated with cisplatin first, then cultured in the presence or absence of LPS in the culture. The cells were harvested at time points of 24, 48, 72 and 96 h, respectively, and analyzed by RT-qPCR. The results showed that FasL mRNA was detected in the cells that maintained stable until 48 h post culture; since then, the FasL mRNA levels declined spontaneously in both NC cells and LC cells, which was counteracted by the presence of LPS in NC cells, but not in LC cells (Fig 2A and 2B). The effects of LPS were abolished by depleting the TLR4 expression (Fig 2B and 2C). The results indicate that FasL mRNA decays spontaneously in NC cells and LC cells, which can be counteracted by the presence of LPS in NC cells, but not in LC cells. The results suggest that activation of TLR4 can maintain the FasL mRNA levels in NC cells.

**Fig 2:** FasL mRNA decays spontaneously. NC cells and LC cells were exposed to cisplatin in the culture for 48 h to increase the expression of FasL, washed with fresh medium, and then cultured in the presence or absence of LPS (100 ng/ml). The cells were harvested at indicated timepoints and analyzed by RT-qPCR. The curves show the levels of FasL mRNA in LC cells (A) and NC cells (B). C, results of TLR4 RNAi. TLR4d: TLR4-deficient NC cells. #, TLRd NC cells exposed to LPS in the culture. Data are presented as mean ± SEM and represent 6 independent experiments.

### Mal expression is impaired in lung epithelial cells of LC patients

We then check the major components of the signal transduction pathway of TLR4 in NC cells and LC cells. The results showed that the expression of TLR4 and MyD88 was not significantly different between NC cells and LC cells, while the Mal levels were significantly lower in LC cells as compared to that in NC cells (Fig 3). The results suggest that the Mal expression impairment may be associated with the FasL mRNA decay in LC cells.

**Fig 3:** LC cells express less Mal. LC tissue was collected from LC patients (n = 18). LC cells and NC cells were isolated and analyzed by RT-qPCR and Western blotting. A-B, levels of TLR4. C-D, levels of MyD88. E-F, levels of Mal. Data of bars are presented as mean ± SEM. Each dot in bars presents data obtained from one sample. Statistics: *t* test.

### Mal expression impairment is associated with FasL mRNA decay in LC cells

Data of Figs 2 and 3 imply that the Mal expression impairment may be associated with the FasL mRNA decay in the cells. To test this, NC cells were treated with Mal RNAi to knock down the expression of Mal (Fig 4A). Mal-insufficient NC cells were treated with cisplatin first to up regulate FasL expression [18] and then cultured in the presence or absence of LPS for 48 h. The results showed that FasL mRNA decay was observed in NC cells 48 h post culture that was counteracted by the presence of LPS; such an effect was abolished in Mal-deficient NC cells (Fig 4B). On the other hand, LC cells were transfected with Mal-expressing plasmids to reconstitute the Mal expression (Fig 4C). Indeed, reconstitution of Mal stabilized the expression of FasL in the cells in the presence of LPS in the culture (Fig 4D). The results pinpoint the importance of Mal in stabilization of FasL expression in LC cells.

**Fig 4:** Mal deficiency is associated with FasL mRNA decay. A-B, NC cells were prepared and exposed to cisplatin in the culture for 48 h. The cells were then washed with fresh medium and treated with Mal RNAi to knock down Mal expression (A). The cells were cultured in the presence or absence of LPS (100 ng/ml) for 48 h. The bars indicate the levels of FasL mRNA (B). C-D, LC cells were prepared; the cells were transfected with Mal-expressing plasmids or control plasmids to restore the expression of Mal (C). The cells were exposed to cisplatin in the culture for 48 h to up regulate the expression of FasL. After washing with fresh medium, the cells were cultured in the presence or absence of LPS (100 ng/ml) for 48 h. The bars indicate the levels of FasL mRNA in the cells. Data of bars are presented as mean ± SEM. Each dot in bars presents data obtained from one sample. Statistics: *t* test.

### Mal induces TDP-43 expression to stabilize FasL expression

Published data indicate that TDP-43 can stabilize some mRNAs by physical contact [19]. We wondered if TDP-43 played a role in stabilizing FasL mRNA in LC cells. To this end, we assessed TDP-43 expression in LC cells and NC cells. The results showed that TDP-43 expression was significantly lower in LC cells than that in NC cells (Fig 5A and 5B). A positive correlation was identified between expression of TDP-43 and Mal in the cells (Fig 5C and 5D). The results imply that Mal activation may increase TDP-43expression. To test this, NC cells were exposed to LPS in the culture for 48 h. The results showed that LPS up regulated TDP-43 expression in the cells, which was abolished by knocking down Mal expression by RNAi (Fig 5E and 5F). We further identified a complex of TDP-43 protein and FasL mRNA in NC cells, the amounts of which were markedly less in LC cells (Fig 5G and 5H). In addition, knockdown of TDP-43 expression significantly reduced the FasL mRNA levels in NC cells (Fig 5I and 5J), while restoration of TDP-43 increased FasL mRNA levels in LC cells (Fig 5K and 5L). The results demonstrate that activation of Mal can modulate TDP-43 expression in NC and LC cells.

**Fig 5:** Activation of Mal modulates TDP-43 expression. A-B, lung cancer (LC) tissue was collected from LC patients (n = 18). LC cells and NC cells were isolated from the tissue and analyzed by RT-qPCR and Western blotting. Bars indicate the levels of TDP-43 mRNA (A) and immunoblots indicate TDP-43 protein (B). C-D, scatter dot blots indicate a positive correlation between TDP-43 and Mal in NC and LC cells. E-F, NC cells were cultured in the presence of LPS at indicated concentrations (denoted on the x axis of E) for 48 h. Bars indicate the mRNA levels of TDP-43. Immunoblots indicate the protein levels of TDP-43. G-H, HC cells and LC cells were prepared and analyzed by RNA-immunoprecipitation assay; a complex of FasL mRNA and TDP-43 protein was identified. Bars indicate FasL mRNA in the complex. Immunoblots indicate TDP-43 protein in the complex. I, results of TDP-43 RNAi. J, NC cells (with or without TDP-43 depletion) were exposed to cisplatin in the culture for 48 h. Bars show FasL mRNA expression in EC cells. K, results of TDP-43 restoration by transfection of TDP-43 expressing plasmids (TDP-43R). L, Bars show FasL mRNA expression in LC cells. Data of bars are presented as mean ± SEM. Each dot in bars presents data obtained from one sample. Statistics: A and G, *t* test. E, ANOVA: p<0.0001; *p<0.01, compared with the group “0” (Bonferroni test). J and L, ANOVA + Dunnett’s test. Data of B represent 6 independent experiments (protein extracts of 18 samples were pooled). Data E-H represent 6 independent experiments. #, cells were treated with Mal RNAi to knock down the expression of Mal. $, cells were treated with control RNAi.

### Reconstitution of Mal restores apoptotic machinery in LC cells

The results of Fig 5 imply that the physical contact of TDP-43/FasL mRNA may play a role in regulation of apoptosis in the cells. To test this, we knocked down TDP-43 or FasL in NC cells by RNAi. The cells were exposed to cisplatin in the culture for 48 h. The results showed that knockdown either TDP-43 or FasL significantly reduced the number of apoptotic cells (Fig 6A and 6B). On the other hand, we reconstituted Mal expression in LC cells by transfection with Mal-expressing plasmids. The cells were exposed to LPS and cisplatin in the culture for 48 h and analyzed by flow cytometry. The results showed that exposure to cisplatin induced markedly more apoptotic cells in those reconstituted with Mal-expressing plasmids as compared to those transfected with control plasmids (Fig 6C and 6D). The results demonstrate that reconstitution of Mal can restore apoptotic machinery in LC cells. Taking together, the results show that deficiency or insufficiency of Mal may impair TDP-43 expression and result in less complexes of TDP-43/FasL mRNA complexes to induce defects of apoptosis in the cells.

**Fig 6:** Restoration of apoptotic machinery in LC cells by modulation of Mal or TDP-43 expression. A-B, NC cells were prepared and treated with Mal RNAi or TDP-43 RNAi to knock down the expression of Mal or TDP-43. The cells were exposed to cisplatin in the culture for 48 h. The gated dot plots show apoptotic cells. The bars show summarized data of apoptotic cells. C-D, LC cells were prepared and transfected with Mal-expressing or TDP-43-expressing plasmids as denoted above each subpanel. The cells were exposed to cisplatin in the culture for 48 h. The gated dot plots show apoptotic cells. The bars show summarized data of apoptotic cells. Data of bars are presented as mean ± SEM. Each dot in bars presents data obtained from one sample. The data represent 6 independent experiments. Statistics: ANOVA + Bonferroni test.

## Discussion

The present data show defects of apoptosis in human LC cells. Defects of apoptosis may be attributed to FasL mRNA decays that occurs spontaneously in the cells. FasL mRNA decay can be blocked by the presence of LPS in the culture, suggesting that activation of TLR4 and its signal transduction pathway can prevent FasL mRNA decay in the cells. Further evidence shows that Mal activation increases TDP-43 expression, the latter physically contacts FasL mRNA to prevent it from decay.

The data show that LC cells have the defects of apoptosis, a phenomenon of apoptosis deregulation [20]. Apoptosis is an important physiological phenomenon in the cell. Deregulation of apoptosis may result in cancer cell over growth to develop into cancer, or induce apoptosis resistance in cancer cells [21]. We used cisplatin to induce apoptosis in experiments. Less LC cells were in a state of apoptosis. The data show that exposure to LPS stabilize FasL. Cisplatin is a drug extensively used in the anti-cancer therapy. The data suggest that LC cells naturally have apoptosis resistance.

In this study, we found that the amounts of FasL mRNA could be up regulated by exposing to cisplatin in both NC cells and LC cells. The fact indicates that the gene transcription of FasL is at functional status in both NC cells and LC cells. The data also show that the FasL mRNA decays spontaneously in both NC cells and LC cells. The presence of LPS can counteract the FasL mRNA decay in NC cells, but not in LC cells. Such a phenomenon suggests that the TLR4 signal is required in the stabilization of FasL mRNA in the cells. This is also noted in the other research system; such as Tian et al reports that activation of TLR4 regulates the FasL/caspase pathway in the liver graft survival [22]. By screening several components of the TLR signal transduction pathway, we found that Mal expression was low in LC cells as compared to that in NC cells. Mal is an important signal adaptor protein in the signal transduction pathway of TLR4 activation, and is required for TLR4-induced myddosome assembly [23]. Our data add novel data to Mal study that Mal is also involved in the induction of TDP-43 expression in LC cells. The data show that exposure to LPS stabilizes FasL mRNA in NC cells but not in LC cells because the deficiency or insufficiency of Mal in LC cells. As LC cells were isolated from the surgically removed LC tissues, LC patients had not received any anti-cancer therapies, the deficiency of Mal in LC cells may contribute to the pathogenesis of LC.

FasL is mainly expressed in T cells and natural killer cells. By activating Fas on target cells, FasL induces target cell apoptosis [24]. In this study, we found that LC cells and NC cells also expressed FasL in response to cisplatin. Such a phenomenon was also found by An et al that airway epithelial cells express FasL upon exposure to 3-methyl-4-nitrophenol, a component of diesel-exhaust particles; the endogenous FasL induces epithelial cell apoptosis [25]. A similar event was found in CD4^+^ T cells. He et al reported that FasL expression was increased in CD4^+^ T cells upon poly clonal activation that induced CD4^+^ T cell apoptosis [26]. Like previous studies [18], we also induced FasL expression in NC cells by exposure to cisplatin in the culture that induced NC cell apoptosis. Because of less amounts of FasL could be induced in LC cells, exposure to cisplatin unable to induce LC cell apoptosis in the culture, a phenomenon like apoptosis resistance occurs in cancer under chemoradiotherapy [27]. We observed that levels of caspase 3 and 8 were not altered in the cells after exposing to cisplatin, this is inconsistent with previous reports [28]; whether are alternative apoptotic pathways activated? This needs to be further investigated.

The data show that activation of Mal up regulates the TDP-43 expression in NC cells and LC cells. TDP-43 is a DNA- and RNA-binding protein [15] and associates with the pathogenesis of cancer [16]. Our data show that TDP-43 bound FasL mRNA in NC cells and LC cells, but the amounts of TDP-43 and TDP-43/FasL mRNA complexes are less in LC cells. Such a feature in LC cells is associated with the lower levels of FasL mRNA in LC cells. We may envisage a scenario that less signal of Mal results in less expression of TDP-43. Because of TDP-43 is required to protect FasL mRNA from decay, the less amounts of TDP-43 results in FasL mRNA decay, and thus, develops apoptosis resistance in the cells. On the other hand, previous reports indicate that the transmembrane activator, calcium modulator, and cyclophilin ligand interactor (TACI) receptor can regulate T-cell-independent marginal zone B cell responses through innate activation-induced cell death [29]. Whether TDP-43 also participates TACI receptor activities in regulating apoptosis is to be investigated.

In summary, the present data show that LC cells have defects of apoptosis that attributes to FasL mRNA decay. The insufficiency of Mal expression in LC cells results in less amounts of TDP-43 expression, the latter is required in stabilization of FasL mRNA in LC cells. Reconstitution of TDP-43 expression in LC cells restores the sensitiveness to apoptosis inducers that may develop to a novel anti-cancer therapy.

## Supporting information

S1 Fig Apoptosis related activities in NC and LC cells. NC cells and LC cells were prepared as described in the text as well as denoted on the x axis. A-C, bars show the mRNA levels of Fas (A), p53 (B) and Bcx (C) in NC cells and LC cells. D-E, bars indicate the activities of caspase (casp) 3 and caspase 8 in NC cells and LC cells. Data of bars are presented as mean ± SEM. Each dot in bars presents data obtained from one sample. NC: Normal control. LC: Lung cancer. Statistics: ANOVA.
(DOCX)

S2 Fig Full-length gel photographs of this paper. (PDF)
